# Efficacy and Safety Analysis of Submucosal Tunnel Endoscopic Resection for Submucosal Masses in Esophageal Muscularis Propria

**DOI:** 10.1155/2022/4457696

**Published:** 2022-09-26

**Authors:** Qianyi Liu, Weishan Ruan, Zhishang Liu, Jiefeng Li, Jiayan Li

**Affiliations:** Department of Gastroenterology, Zhongshan City People's Hospital, Zhongshan 528400, Guangdong Province, China

## Abstract

**Objective:**

To analyze the efficacy and safety of submucosal tunnel endoscopic resection (STER) for the treatment of submucosal masses in esophageal muscularis propria.

**Method:**

A total of 272 patients with submucosal masses in esophageal muscularis propria diagnosed and treated in our hospital from February 2019 to January 2022 were randomly selected for the study and then were randomly divided into the STER group (*n* = 136) and the endoscopic mucosal dissection (ESD) group (*n* = 136) according to the random number table method. Patients in the STER and ESD groups were treated with STER and ESD, respectively. The clinical data of patients from the two groups were collected and compared. The clinical effects and the changes of surgery-related indexes of patients after ESD and STER treatment were observed. The safety of ESD and STER was compared. The factors influencing the efficacy of STER treatment for submucosal masses in esophageal muscularis propria were analyzed.

**Result:**

There were significant differences between the STER group and the ESD group in terms of tumor size, lesion level, adhesion and surgical approaches (*P* < 0.05). The effective rates of ESD treatment and STER treatment were 98.53% and 88.97%, respectively. Meanwhile, the effective rates of STER treatment were significantly higher than those in the control group (*P* < 0.05). In addition, the patients in the STER group had longer operation time, less blood loss, and shorter hospital stay compared with those in the ESD group (*P* < 0.05). Adverse reactions occurred during ESD treatment and STER treatment included delayed bleeding, adhesion, perforation, and pleural effusion with the total incidence of adverse reactions of 4.41% and 13.97%, respectively. The adverse reactions in STER group were prominently less than these in the ESD group (*P* < 0.05). Logistic multivariate regression analysis showed that independent risk factors, including tumor size, lesion level, adhesion, and surgical approaches, affected the efficacy of STER in the treatment of submucosal masses in esophageal muscularis propria (*P* < 0.05).

**Conclusion:**

STER is an effective method for the treatment of submucosal masses in esophageal muscularis propria, which can exhibit a good effect with faster postoperative recovery and higher safety, thereby being worthy of clinical application and promotion. Tumor size, lesion level, adhesion, and surgical approaches are all related factors affecting the effect of STER treatment.

## 1. Introduction

Submucosal masses in esophageal muscularis propria is a kind of tumor that originated from the mucosal layer of the esophageal proper muscularis, which usually does not cause clinical symptoms. Most of them are benign lesions, and a few are gastrointestinal stromal tumors with malignant potential. As the tumor continues to grow, it will compress the surrounding organs, causing difficulty in breathing. Additionally, if the tumor has malignant features such as ulcers and erosions, it will manifest as gastrointestinal bleeding, hematemesis, and melena. With the continuous progress of medical technology, the diagnosis and diagnosis rate of diseases are gradually increasing. Due to the submucosal masses located in the esophageal muscularis propria, it is easily overlooked, thus delaying the treatment time. Surgery is the main method for the treatment of submucosal masses in esophageal muscularis propria and the main approach for diagnosing whether the disease is malignant [1, 2]. The traditional open surgery used in the past clinically not only causes greater trauma to the patient but also has a high recurrence rate after surgery, which seriously affects the patient's life [3].

With the rapid development of minimally invasive technology and endoscopic treatment technology, endoscopic treatment has gradually been widely used in clinical practice and has been recognized by people due to its advantages of less trauma to patients and shorter postoperative recovery time. Submucosal tunneling endoscopic resection (STER) is a resection treatment mainly used for the upper gastrointestinal mucosa originating from the muscularis propria. By establishing a submucosal tunnel to remove the lesions, the integrity of the mucosa can be effectively maintained and the incidence of perforation can be reduced. During the STER process, the vascular network of the wound can be clearly displayed, which greatly reduces the bleeding caused by accidental cutting of blood vessels. Additionally, the operation of STER in the esophageal cavity can avoid the free operation of the peripheral mediastinum structure of the esophagus and reduce the possibility of damage to the tissue structure [4]. It has been reported that STER has achieved good results in the treatment of rectal carcinoid, and there is no residual disease or disease recurrence after surgery and no serious complications with a good effect [5]. However, its effect on the submucosal masses in esophageal muscularis propria remains unclear.

In this study, patients with submucosal masses in esophageal muscularis propria who were diagnosed and treated in our hospital from 2019 to 2022 were selected as the research subjects, and they were randomly divided into two groups treated with ESD and STER, respectively. The study was aimed at investigating the efficacy and safety of STER in the treatment of diseases.

## 2. Materials and Methods

### 2.1. General Materials

A total of 272 patients with submucosal masses in esophageal muscularis propria diagnosed and treated in our hospital from February 2019 to January 2022 were selected as the research subjects by a randomized, double-blind method. There were 150 males and 122 females, aged 26-72 years, with an average age of 51.58 ± 5.29 years. The following are the inclusion criteria: (1) patients with esophageal submucosal masses found through imaging detection, (2) patients with benign lesion verified through pathological examination, (3) patients with intact mucosa, (4) patients who had signed the informed consent form and actively participated in the study, (5) patients with complete clinical and pathological data and could cooperate with the study, and (6) patients over 20 years old. The following are the exclusion criteria: (1) patients with malignant lesions or distant metastasis of tumors, (2) patients with obviously abnormal liver and kidney function or heart function, (3) patients with abnormal coagulation function, (4) patients who were intolerant to surgery, and (5) patients in pregnant or lactating stage. A total of 272 patients with submucosal masses in esophageal muscularis propria were randomly divided into the STER group and the ESD group according to the random number table method, with 136 patients in each group. According to whether the treatment was effective or not, the patients were divided into an effective group and an ineffective group, including 255 cases in the effective group and 17 cases in the ineffective group. All the studies were approved by the Clinical Research and Laboratory Animal Ethics Committee of Zhongshan People's Hospital (approval number: K2020-107). The general data selection is displayed in Figure 1.

### 2.2. Methods

#### 2.2.1. The ESD Group

The patients in the ESD group were treated with ESD. Blood routine examination and electrocardiogram were performed before operation. The patient was placed in lateral position and given intravenous anesthesia. The size and location of the lesion were determined by indigo carmine staining, and the lesion was marked at the edge of the lesion. 2.5 mL of indigo carmine was mixed with an appropriate amount of adrenaline in normal saline and injected at the lesion and edge marking points with the multipoint injection to make the mucosa fully uplift. The mucosa outside of the mark was completely cut open with a hook knife and dissection to ensure complete excision of the lesion with the use of coagulation or heat forceps for hemostasis. The patients underwent postoperative fasting and infection prevention and were closely monitored with vital signs.

#### 2.2.2. The STER Group

The patients in the STER group were treated with STER. The size and location of lesions were confirmed by using endoscopic ultrasonography before surgery, and the patients were fasting before surgery. The patients were placed in a lateral position and administered with intravenous anesthesia. The esophagus was flushed with normal saline, and a mixture of indigo carmine and adrenaline in normal saline was injected for labeling. The upper and lower mucosal layers were separated, the mucosal layer was incised, a submucosal tunnel was established at a distance of about 1.5 cm from the tumor until the tumor was completely exposed, and the lesions were excavated. The tumor was separated from the muscularis propria of the esophagus, the tumor was taken out, the tunnel was flushed with sterile saline, the bleeding was stopped using electrocoagulation or thermal forceps, and the tunnel was clamped with titanium clips. The patients underwent postoperative fasting and were strictly monitored with vital signs and with postoperative antibiotics for anti-infection (Figure 2).

### 2.3. Clinical Pathological Data Collection

The clinical pathological data of patients were collected, including the age (≤45 years old, >45 years old), gender (male, female), tumor size (≤6 cm^3^, >6 cm^3^), pathological type (lipoma, leiomyoma, granulosa cell tumor, and stromal tumor), pathological level (nonintrinsic muscle layer, intrinsic muscle layer), location of onset (upper 1/3 of esophagus, middle 1/3 of esophagus, and lower 1/3 of esophagus), adhesion (yes, no), and surgical method (STER, ESD).

### 2.4. Outcome Measures

#### 2.4.1. Efficacy Analysis

Endoscopy review was performed 6 months after treatment [6], including deterioration, stability, partial remission, and complete remission. Among them, manifestations that the volume of the lesions increased by more than 30% or new lesions were appeared after treatment was regarded as deterioration; manifestations that the volume of lesions decreased by less than 30% after treatment and did not reach the degree of deterioration was regarded as stable; manifestations that the volume of lesions decreased by more than 30% after treatment was regarded as partial remission; manifestations that lesions were complete obliteration was regarded as complete remission. Total effective rate of treatment = (stability + partial remission + complete remission)/total number of cases × 100%.

#### 2.4.2. Detection of Operation-Related Indexes

The changes of indexes, including the operation time, intraoperative blood loss, and hospitalization time of ESD and STER in the treatment of submucosal masses in esophageal muscularis propria were recorded.

#### 2.4.3. Safety Analysis

Adverse reactions, including delayed bleeding, adhesion, perforation, and pleural effusion, were recorded in the treatment of submucosal masses in esophageal muscularis propria, to compare the safety of ESD and STER treatment.

#### 2.4.4. Analysis of Influencing Factors

The two groups of patients were divided into an effective group and an ineffective group according to the treatment effect, and the influencing factors of the effect of STER in the treatment of submucosal masses in esophageal muscularis propria were analyzed.

### 2.5. Statistical Analysis

The data were analyzed using SPSS 21.0 statistical software. Enumeration data, such as the univariate analysis of the efficacy and safety of STER in the treatment of submucosal masses in esophageal muscularis propria, were expressed as cases (%) and compared with the *χ*^2^ test or Fisher's exact test. Measurement data, such as operation time, blood loss, and hospitalization time, were tested by normal distribution, which were in line with normal distribution. Measurement data were expressed as $\bar{x}\pm s$ and compared using a *t*-test. *P* < 0.05 indicated that the difference was statistically significant.

## 3. Results

### 3.1. Comparative Analysis of Clinical Data

There were no significant differences in age, gender, pathological type, and location of the disease between the STER group and the ESD group (*P* > 0.05), while significant differences were discovered in tumor size, lesion level, adhesion, and surgical approaches (*P* < 0.05) (Table 1).

### 3.2. Analysis of the Curative Effect of STER in the Treatment of Submucosal Masses in Esophageal Muscularis Propria

The effective rates of ESD treatment and STER treatment were 98.53% and 88.97%, respectively, The effective rates in the STER group were significantly higher than those in the ESD group (*P* < 0.05). (Table 2).

### 3.3. Comparison of Surgical Related Indexes in the Treatment of Submucosal Masses in Esophageal Muscularis Propria

Compared with those in the ESD group, the operation time was significantly prolonged, the bleeding volume was observably reduced, and the hospitalization time was notably shortened in the STER group (*P* < 0.05) (Table 3).

### 3.4. Safety Analysis of STER in the Treatment of Submucosal Masses in Esophageal Muscularis Propria

Adverse reactions that occurred during ESD and STER treatment included delayed bleeding, adhesions, perforation, and pleural effusion. The incidences of adverse reactions in the ESD groups were 0.74%, 3.68%, 2.21%, and 5.15%, severally, while these in the STER groups were 0.74%, 2.21%, 0.74%, and 2.94%, respectively. The total incidence of adverse reactions in the two groups was 4.41% and 13.97% separately, which was significantly lower in the STER group than in the ESD group (*P* < 0.05). (Table 4).

### 3.5. Multivariate Analysis of the Effect of STER in the Treatment of Submucosal Masses in Esophageal Muscularis Propria

The indicators with significant differences in univariate analysis were selected for logistic multivariate regression analysis. The results showed that tumor size, lesion level, adhesion, and surgical approaches were all independent risk factors affecting the efficacy of STER in the treatment of submucosal masses in esophageal muscularis propria (*P* < 0.05) (Table 5).

## 4. Discussion

Submucosal masses in esophageal muscularis propria is a relatively rare esophageal tumor in clinic. According to relevant statistics, submucosal masses in esophageal muscularis propria accounts for only about 1% of all esophageal tumors. However, most lesions in submucosal masses in esophageal muscularis propria have no obvious clinical symptoms with the manifestation of dysphagia, which leads to missed diagnosis, misdiagnosis, and delayed treatment [7, 8]. The pathological types of submucosal masses in esophageal muscularis propria include lipoma, leiomyoma, granulosa cell tumor, and stromal tumor. Among them, leiomyoma and stromal tumor are more common. Moreover, stromal tumors have a certain potential of malignant advance. The larger the volume is, the higher the degree of malignancy and the worse the prognosis is. Therefore, early diagnosis and timely treatment are of great significance. In the past, the clinical diagnosis is mainly based on imaging, endoscopic, and pathological examinations to observe the shape, color, and mobility of the lesions. However, the diagnosis is difficult, because the lesions are located in the submucosal mucosa [9].

With the continuous development of minimally invasive technology, resection of submucosal masses in esophageal muscularis propria by thoracoscopy is gradually applied in clinical practice. However, the application of thoracoscopy in large-area lesions is still immature, because it cannot completely remove the lesions, resulting in a high recurrence rate. ESD is a technology developed on the basis of endoscopic mucosal resection, which has a high success rate in large-area lesion resection and significantly reduces the postoperative recurrence rate. However, ESD is always accompanied with a high perforation and postoperative bleeding rate [10, 11]. The effectiveness and safety of clinical treatment are important factors affecting the promotion and application. In recent years, STER has been gradually developed, which is a method of tumor resection under the submucosal tunnel constructed between the mucosal layer and the muscularis propria. STER is developed based on ESD, but it can maintain the integrity of mucosal layer to the greatest extent, reduce the risk of infection, and prevent the outflow of postoperative fluid [12]. Studies have found that STER has shorter hospitalization time and faster postoperative recovery compared with other endoscopic resection and traditional open surgery [13]. In the study of gastric submucosal tumors, it was found that the combined estimated values of total resection and complete resection of STER were about 95.12% and 97.86%, respectively, and the combined estimated values of gas-related complications, mucosal tear, and delayed bleeding were about 8.72%, 4.20%, and 2.10%, respectively [14]. STER is a safe and effective resection of gastric submucosal tumors with few complications. In the study of gastroesophageal tumors by domestic scholars [15], by analyzing the treatment of STER and endoscopic mucosal tumor excision (ESE), it was shown that STER has a shorter operative time, less pain, less intraoperative blood loss, and faster postoperative recovery compared with ESE. STER is an effective method for the treatment of gastroesophageal muscularis propria tumors. In this study, the efficacy, surgical related indicators, and adverse reactions of ESD and STER in the treatment of submucosal masses in esophageal muscularis propria were compared. It was found that STER treatment had a higher clinical effect, a lower incidence of adverse reactions, an apparently reduced amount of bleeding, and an obviously shorter length of stay, but a longer operation time and a slower operation speed. The reason is that by establishing a tunnel, STER can effectively reduce the wound surface, protect the mucosa at the perforation, and avoid perforation of the pipe wall. Moreover, the muscle layer on the surface of the tumor can be completely stripped to fully expose through the tunnel, so as to quickly and completely peel off and avoid obvious bleeding. However, since STER needs to establish a tunnel and descend slowly, the closer the mucosal surface is, the richer the submucosal blood vessels is, resulting in a longer operation time and slower operation speed [16, 17]. Taken together, STER provides a safe and effective method for the treatment of submucosal masses in esophageal muscularis propria.

In addition, through the analysis about the relevant factors affecting the efficacy of submucosal masses in esophageal muscularis propria, it showed that the size of tumor, lesion level, adhesion, and surgical approaches were all the factors affecting the efficacy of STER in the treatment of submucosal masses in esophageal muscularis propria, and all of them were independent risk factors. Larger tumors generally tend to adopt the traditional treatment method with low treatment cost. Tumors with large volume or growing out of the cavity are difficult to be completely removed from the body, which is a high-risk factor for postoperative adverse reactions of patients [18]. The occurrence of adhesion may increase the pain of patients during the operation and affect the treatment effect. In contrast, the STER tunnel has a large operating space and a clear operating field of view. After the mucosal opening, the submucosa and the muscularis propria are separated, and a tunnel structure is formed between the submucosa and the muscularis propria. The tumor is removed under the tunnel, which can effectively prevent the injury caused by the operation during the operation [19].

In general, STER is an effective method for the treatment of submucosal masses in esophageal muscularis propria, which can have a good effect with faster postoperative patients recover and higher safety, which is worthy of clinical application and promotion. The size of the tumor, the level of the lesion, adhesion, and surgical approaches are all related factors that affect the therapeutic effect of STER. Nevertheless, there are still some limitations in this study. Compared with ESD, the STER technology is not yet fully mature; thus, the early treatment time is relatively long. Additionally, the sample size of the study is small, and the time is still short, which may affect the results. Therefore, more cases and comparative studies confirm the safety and efficacy of this procedure in the following study.

## Figures and Tables

**Figure 1:** The process of general data selection.

**Figure 2:** STER procedure and the follow-up. (a) Large tumor found under esophageal mucosa; (b) incision of esophageal mucosa; (c) tumor exposure; (d) gradual stripping; (e) complete stripping; (f) postoperative follow-up.

**Table 1:** Comparative analysis of clinical data between the STER group and the ESD group [cases (%)].

	The STER group (*n* = 136)	The ESD group (*n* = 136)	$\frac{\chi^{2}}{t}$	*P*
Age (year)			1.075	0.300
≤45	40 (29.41)	48 (35.29)		
>45	96 (70.59)	88 (64.71)		
Gender (%)			0.375	0.540
Male	75 (55.15)	80 (58.82)		
Female	61 (44.85)	56 (41.18)		
Size of the tumor (cm^3^)			66.489	<0.001
≤6	114 (83.82)	48 (35.29)		
>6	22 (16.18)	88 (64.71)		
Pathological type (%)			5.895	0.117
Lipoma	1 (0.74)	0 (0.00)		
Leiomyoma	132 (97.06)	128 (94.12)		
Granulosa cell tumor	2 (1.47)	1 (0.74)		
Stromal tumor	1 (0.74)	7 (5.15)		
Lesion level (%)			77.305	<0.001
Non-intrinsic muscle layer	96 (70.59)	24 (17.65)		
Intrinsic muscle layer	40 (29.41)	112 (82.35)		
Location of onset (%)			4.517	0.104
Upper 1/3 of esophagus	16 (11.76)	8 (5.88)		
Middle 1/3 of esophagus	64 (47.06)	58 (42.65)		
Lower 1/3 of esophagus	56 (41.18)	70 (51.47)		
Adhesions (%)			70.588	<0.001
Yes	4 (2.94)	64 (47.06)		
No	132 (97.06)	72 (52.94)		
Surgical method (%)			66.104	<0.001
STER	37 (27.21)	104 (76.47)		
ESD	99 (72.79)	32 (23.53)		

**Table 2:** Efficacy analysis of STER in the treatment of submucosal masses in esophageal muscularis propria [cases (%)].

Groups	Cases	Complete remission	Partial remission	Stability	Deterioration	Effective rate
The STER group	136	56 (41.18)	70 (51.47)	8 (5.88)	2 (1.47)	134 (98.53)
The ESD group	136	49 (36.03)	59 (43.38)	13 (9.56)	15 (11.03)	121 (88.97)
*χ* ^2^		0.760	1.784	1.290	10.604	10.604
*P*		0.383	0.182	0.256	0.001	0.001

**Table 3:** Comparison of surgical related indexes for the treatment of submucosal masses in esophageal muscularis propria ($\bar{x}\pm s$).

Groups	Cases	Operative time (min)	Operation speed (mm^2^/min)	Bleeding volume (mL)	Length of stay (d)
The STER group	136	66.38 ± 18.13	2.73 ± 0.68	2.63 ± 0.52	3.74 ± 0.42
The ESD group	136	46.24 ± 15.47	3.95 ± 0.71	4.78 ± 1.26	6.50 ± 0.74
*t*		9.855	14.472	18.394	37.858
*P*		<0.001	<0.001	<0.001	<0.001

**Table 4:** Safety analysis of STER in the treatment of submucosal masses in esophageal muscularis propria [cases (%)].

Groups	Cases	Delayed bleeding	Adhesion	Perforation	Pleural effusion	Total cases
The STER group	136	1 (0.74)	3 (2.21)	1 (0.74)	1 (0.74)	6 (4.41)
The ESD group	136	5 (3.68)	7 (5.15)	3 (2.21)	4 (2.94)	19 (13.97)
*χ* ^2^		2.727	1.661	1.015	1.834	7.444
*P*		0.099	0.197	0.314	0.176	0.006

**Table 5:** Multivariate analysis of the effect of STER in the treatment of submucosal masses in esophageal muscularis propria.

Factors	Regression coefficient	Standard error	Wald value	*P* value	Odds ratio	95% confidence interval (CI)	
						Lower limit	Upper limit
Size of the tumor	1.287	0.531	5.150	0.023	3.571	1.414	9.505
Lesion level	1.839	0.514	10.056	<0.001	7.245	2.048	12.015
Adhesions	1.319	0.526	6.468	0.008	4.867	1.368	10.016
Surgical approach	1.505	0.615	5.591	0.018	4.023	1.268	11.520

## Data Availability

The datasets used and/or analyzed during the current study are available from the corresponding author on reasonable request.
